The article "Research on Children's Cognitive Education Based on Pathological Linguistics" was published in 2022. Journal: Occup Ther Int.

# Research on Children's Cognitive Education Based on Pathological Linguistics

**DOI:** 10.1155/2022/8692238

**Published:** 2022-08-04

**Authors:** Yuefang Hou

**Affiliations:** Lvliang University, Lvliang, Shanxi 033000, China

## Abstract

The value of pathological linguistics in children's cognitive development has attracted more and more experts' attention. Based on pathological linguistics, this paper establishes an intervention system for children's cognition-language assessment and cognitive education, guided by a set of fixed procedures, which can quickly collect children's speech data in a short period of time. Based on this evaluation paradigm, the lab collected a large number of speech data of children aged 2-14 in the process of verbal communication. Based on the six linguistic dimensions of phonology, productivity, fluency, grammar, semantics, and logic, the corpus was subdivided into 16 indicators for manual annotation and machine recognition. A cognitive-language assessment database is established for language ability assessment and language barrier screening, and on this basis, the children's language assessment and cognitive education intervention system is completed based on six modules: user, assessment, scale, resources, teaching, and data. Through experimental research, this paper proves that there are differences in the contribution rates of six language dimensions to the screening of children's language disorders, and the top three are fluency (29.6%), pronunciation (25.7%), and productivity (19.3%). By analyzing the contribution rates, the development of children's comprehensive speech ability can be evaluated more accurately. The early intervention education of children's cognition has a great relationship with their comprehensive language ability. The intervention education before the age of 3 is beneficial to the language development of children with disabilities. Children's cognitive education has improved in cognitive performance, cognitive generalization level, emotional cognition, and language expression, indicating that the use of cognitive education system has a good effect, improving the level of children's cognitive education.

## 1. Introduction

As an important force of national development, children's healthy growth is crucial. Children's cognitive education has been paid more and more attention by all walks of life. Human cognition is a process of continuous development, rather than being born with familiarity with everything in the world and understanding of things and various situations [1]. Children in different stages, their physical and psychological characteristics and behavior, preferences are also very different. Cognition is a process of continuous development from birth, infant, preschool, and school age to adolescent stage, and each stage has different cognitive performance [2].

The article "Research on Children's Cognitive Education Based on Pathological Linguistics" was published in 2022. Journal: Occup Ther Int.

Language is the most important tool for cognition of the world. In children's cognitive education, language is the only feasible way to help children understand the world. In the process of children's cognitive development, language communication is the most important cognitive channel, very important to children, great influence. However, in the process of language acquisition, children often have various obstacles, defects, or disorders due to various reasons, which directly affect children's cognitive education and intellectual development, leading to psychological changes [3]. Therefore, children's language disorder has been the focus of many scholars and experts. In view of children's language disorders, neurolinguistics explores the pathological mechanism of language disorders from different aspects and professional perspectives and uses various means to diagnose and treat language disorders.

With the development of society and the improvement of education level, children's cognitive education informational has become the development trend. The background of traditional manual intervention methods is psychology, and the background of other disciplines is relatively lacking. It can be seen that the interdisciplinary research on children's cognitive education is very weak, so it is necessary to strengthen the cooperative research among various disciplines, such as linguistics, medicine, rehabilitation, psychology, and special education. The evaluation and intervention system for children's cognitive education based on pathological linguistics has achieved multidisciplinary research and has broad prospects for development [4]. This system establishes an intervention system for children's language assessment and cognitive education from the perspective of pathological linguistics. The system can predict and evaluate the basic situation of children's cognitive development, providing basic data and intervention direction for cognitive education intervention.

## 2. Related Discussion

Cognitive education belongs to heuristic education, which means that in order to achieve a certain educational goal, educators use educational means to help the educates to build up their perception, attention, and thinking ability of a learning skill from the perspective of cognitive psychology [5]. The development of children's cognitive education is inseparable from the study of children's cognitive theory. In the 1960s, modern cognitive theory expanded and enriched the theory of children's cognitive development, which brought great influence to the research of children's cognitive development. Thojampa put forward the theory of epistemology and children's psychological development stage and systematically and fully discussed the mechanism of children's cognitive development and the characteristics of children's psychological development at different ages, laying a solid theoretical basis for modern children's cognitive education research [6]. Syahputri's research on children's development and educational psychology is also quite rich. He believes that environment, language, and education are the three major factors affecting children's psychological development. Rezyana inherited and developed previous theoretical studies and mainly studied children's moral cognition and judgment ability [7]. In addition, both children's cognitive development theory and modern cognitive psychology have mentioned information processing psychology. Perales and Baxter described the information processing mode and its four stages completely, which played a significant guiding role in studying children's specific cognitive process [8].

The article "Research on Children's Cognitive Education Based on Pathological Linguistics" was published in 2022. Journal: Occup Ther Int.

The theory of cognitive education holds that children's cognition is a process of continuous development and change, and language ability is one of the most important characteristics of cognitive development. In the process of children's continuous growth, language barriers will occur because of various physiological and psychological reasons. Pathological linguistics is the application of theories and methods in various medical disciplines and linguistic fields to study, diagnose, and treat various types of language disorders, defects, or disorders, with strong experimental and great application value [9]. Pathology started in the 1920s, and speech pathology was first established by Carl Emil Seashore, who studied sound and hearing [10]. In 1925, the American Society of Speech Correction was established in the United States [11]. In recent years, more and more attention has been paid to linguistics. Researchers and clinicians have realized that the correct understanding and accurate analysis of language disorders can only be realized by linguistic theories and the concepts and analytical methods of linguistics and its branches. Bob placed language disorders at the core and believed that the task of pathological linguistics is to study the impairment of language ability. Speech, voice, and fluency disorders have nothing to do with language, but represent various impairments in the process of language transmission [12]. Data from a large number of clinical subjects have demonstrated that these subdisciplines of pathology can be used to describe and analyze the characteristics of language disorders.

The article "Research on Children's Cognitive Education Based on Pathological Linguistics" was published in 2022. Journal: Occup Ther Int.

With the development of computer-aided instruction and mobile devices, software has been used for children's cognitive education by virtue of the advantages of computer-aided training. For example, “Baron-friendly English Flash Cards by No Yo” simulates more than 10 scenarios such as “family” and “school” to train cognitive and language skills [13]. Smithers combines cognition and play to attract children to complete interactive responses [14]. Yulduz and Maftuna used the Junior Detective Training Program to train children's emotional cognition, social skills, and understanding [15]. Shulamit used Find Me to train basic social skills [16]. Although the existing applications play the advantages of computer-aided training to some extent, they still cannot meet the development needs of current cognitive education due to the particularity of children's cognitive education. In recent years, the value of pathological linguistics in clinical diagnosis and treatment has been paid more and more attention by experts. People began to explore the development of children's cognitive education based on pathological linguistics.

### 2.1. Construction of Children's Cognitive Education System

Language is an essential communication tool for human beings and a core ability to be acquired in children's cognition [17]. It should be the top priority of cognitive education for children to carry out extensive language ability assessment and accurately screen out children's language disorders as soon as possible. On the basis of assessment, further intervention education on children's cognition is the ultimate goal of promoting the healthy development of children's cognition.

### 2.2. Cognitive Language Assessment Database

This study designed a set of children's cognitive-speech assessment database for language barrier screening, which can quickly assess children's verbal communication level in a short time and then reflect children's cognitive status. Based on this paradigm, we collected a large number of verbal communication data of children aged 2-14, analyzed and labeled the data with six linguistic dimensions and 16 subdivided indicators, and established a cognition-speech database for children that can be used for language ability assessment and language barrier screening.

#### 2.2.1. Fixed Bootstrap

The speech assessment method designed in this paper for language barrier screening for children firstly presents the assessment task to children in the form of pictures, videos, and audio, which is more interesting. During the process, children's speech recordings are collected.  Figure 1 shows the schematic diagram of picture, audio, and video test topics. Secondly, in order to achieve the screening, classification, and grading of language disorders, it is necessary to make a horizontal comparison of the corpus of different speakers. Therefore, the whole set of assessment is guided by a set of fixed procedures to achieve the characteristics of multiple children's speech samples that can be compared. Furthermore, considering that children are prone to distraction, we controlled the number of questions and could quickly and fully guide the optimal speech performance of children in about 10 minutes. Follow the principle of "from easy to difficult" in the evaluation program, collect real and rich data on children's vocabulary, and then evaluate children's language communication ability.

The article "Research on Children's Cognitive Education Based on Pathological Linguistics" was published in 2022. Journal: Occup Ther Int.

#### 2.2.2. Annotation of Corpus

Since children's language disorders have different types, such as hearing and understanding disorders, phonological disorders, and pragmatic disorders; the annotation and scoring of children's speech data should also cover multiple aspects, so as to achieve effective classification and grading of children's language disorders [18]. In terms of database construction, compared with the raw corpus storing the original children's speech data, the carefully and professionally annotated mature corpus is undoubtedly more valuable for research. Therefore, we adopt independent development transfer with software to transfer and multidimensional corpus linguistics manual annotation analysis, and through the machine automatic identification indicators to extract some words (such as pause frequency and duration), including voice, capability, fluency, grammar, semantics, and logic six language dimension, which were divided into 16 indicators. In this way, the children's verbal communication level can be carefully evaluated. Detailed annotation items are shown in Table 1.

In order to ensure the reliability and accuracy of all corpus annotation, we adopted the method of three-round annotation. First of all, two annotators with linguistic expertise are asked to mark the same corpus, respectively. The intuitive scoring should be completely consistent, and the error tolerance rate of all indicators except intuitive scoring should be set at 10%. Then, the corpus with conflicts after two rounds of annotation was selected for annotation for the third time. Three annotators annotated each section of corpus at the same time. If the opinions of the three annotators were still inconsistent after consultation, a voting system was adopted, and finally, the scores of all indicators were obtained. According to the marked data, the CSV format file is automatically generated to further standardize the data result processing. For the negative logic indicators related to voice, fluency, grammar, and logic, the score normalization method is as follows:

(1) $$\begin{array}{c} a^{\prime }=\frac{\left[\max\left(a\right)-a\right]\times \left[\min\left(a\right)+a\right]}{\left[\max\left(a\right)-\min\left(a\right)\right]}, \end{array}$$

where *a* represents the single index score of all subjects' expression data collected by the previous database and *N* represents the number of subjects. For positive logical indicators related to productivity and semantics, the fractional normalization method is as follows:

(2) $$\begin{array}{c} a^{\prime }=\frac{\left[a-\min\left(a\right)\right]\times \left[\max\left(a\right)-a\right]}{\left[\max\left(a\right)-\min\left(a\right)\right]}. \end{array}$$

The normalized score can better represent the ability level of each indicator, and the higher the score is, the stronger the ability is. Annotated data are classified and layered stored in corpus database, which can be used for further data mining, such as big data analysis and machine learning.

The article "Research on Children's Cognitive Education Based on Pathological Linguistics" was published in 2022. Journal: Occup Ther Int.

#### 2.2.3. Establishment of Database

After obtaining the children's original corpus, the first thing to do is to archive the data. Taking the subjects and question types as the unit, the original audio data is classified and stored, and a database of Chinese children's speech communication is established. Second, data alignment is achieved through comprehensive and detailed corpus annotation. Through the collection and annotation of children's corpus, we established a database of children's verbal communication level from 2 to 14 years old. At present, the database has stored the speech data of 966 children under the guidance of fixed procedures. These children come from different levels of economic development, including about 200 ethnic minority children in addition to children, and children include about 200 subjects who master their mother tongue and dialects. About 100 children with language disorders and related diseases (such as hearing impairment, visual impairment, and autism) have abundant data. For these data, we classified and archived them according to subjects and question types and carried out unified text transcriptions. Among them, the corpus of 638 children was annotated and the scores of verbal communication ability were output. The current database overview is shown in Table 2.

The database combined with machine learning technology can be used for intelligent automatic screening of children's language disorders. The corpus guided by fixed program has high comparability, so it is suitable to use machine learning related technology to model training data and realize automatic screening of language disorders. Based on the audio data and annotation data of 284 children's verbal communication level in this database, the dual-channel deep learning algorithm was used to extract the features of speech stream and content stream simultaneously, so as to establish the correlation model between the audio characteristics of children's language, each annotation indicator, and language ability level.

The article "Research on Children's Cognitive Education Based on Pathological Linguistics" was published in 2022. Journal: Occup Ther Int.

### 2.3. Cognitive Education Intervention System

The establishment of children's language assessment database based on pathological linguistics can quickly assess children's verbal communication level and cognitive status in a short time, providing data support for the further construction of children's cognitive education intervention system in this chapter. The system has broad application prospects. At the theoretical level, the general laws of children's language cognition can be explored, and the current children's overall language development profile and the development characteristics of various aspects of language ability can be grasped. At the application level, through comparative analysis, the characteristics of children's cognitive developmental disorders can be found, and the cognitive education development path of special groups can be explored. This has implications for the specific development of the evaluation of children's cognitive impairment in the future.

#### 2.3.1. Structure of Cognitive Education System

See Figure 2. If divided from the function, the system is mainly composed of three layers, namely, the user layer, the application service layer, and the data layer. The user layer is mainly responsible for interacting with users, that is, providing interfaces for different roles to complete corresponding operations. From the point of view of user friendliness, this system adopts the elegant degraded way, compatible with the current mainstream customers, such as Internet Explorer 6 and later versions, Mozilla Firefox, Chrome, 360, Safari, Android client, Pad, and Mac. The application service layer is the core of this system for all business, connecting the user layer and data layer, and is responsible for the communication between the two, limiting the entry of data access; the application service layer in all the modules of the MVC pattern has been adopted for development; when the display content of the layer needs to be updated, we do not need to change or override control layer and data layer, reducing the coupling of system development which is low. It is convenient for program maintenance and version iteration [19]. Data layer, the bottom layer of the system, is also the data warehouse of the system, maintaining all the data required by the system business logic.

The article "Research on Children's Cognitive Education Based on Pathological Linguistics" was published in 2022. Journal: Occup Ther Int.

#### 2.3.2. Cognitive Education System Module

The ultimate goal of pathology is to propose therapeutic strategies for speech disorders and further adjust the results of intervention strategies. The improvement of children's cognitive ability mainly depends on education and behavior intervention. The system can be divided into six modules: user, evaluation, scale, resources, teaching, and data. See Figure 3.

The main functions of these modules are described below.

1. User module: the user module is the most direct module to interact with users. The quality of its design will not only affect the user experience of the system but also restrict some performance of the whole system [20]. In this evaluation system, including the principal, teachers, experts, parents, children, and administrators of six roles, each role has the corresponding user information; in addition to the children role, the other five roles have information registration, user login, information management, and other functions.
2. Assessment module: this is the core module of the self-assessment of the subject, mainly around the assessment of special children's cognition, perception, language communication, and social communication; self-care of these five aspects, because the performance in these five aspects is not normal, is some common characteristics of special children. At present, the system has carefully designed a number of interactive games for statistical analysis of game data.
3. Scale module: it is designed for parents' evaluation. As the guardian of the tested object, parents will have a better understanding of the basic situation of children. In order to facilitate the simplicity and convenience of the parent evaluation module, the system adopts the form of electronic questionnaire and adds a certain interactive effect. In the design of electronic questionnaire, the CARS scale, ABC scale, ASSQ scale, and M-CHAT scale are mainly developed. Finally, through the statistics and analysis of parents' data, we obtain the evaluation results.
4. Resource module is an important module of the system, mainly including children's games, children's animation, children's video, teaching courseware, and teaching tools. It is aimed at meeting the learning needs of children with disabilities who cannot go to school, and pushing learning materials after assessment, and providing relevant resources for staff engaged in special education. In this system, the label is introduced to realize the directional push of resources, and the label is also convenient for resource retrieval. For example, when a parent through the system checked out children in the perception of the possible obstacles, then, the system will automatically take “perception” as a label. Combined with the relevant data of the children, search in the resources, and sort according to the corresponding search heat, utilization rate, time, and other relevant parameters, and then feedback the processed resources to the parents. In the front page, the plug-in Boot Strap-Tagsin PUT is used to simplify the parents' search for relevant learning resources according to the corresponding resource “label”.
5. Teaching module: teaching module is one of the important modules of the system. The module not only creates conditions for teachers to conduct online teaching; at the same time, the module also provides a large number of preschool education video animation, preschool education video, online courseware, teaching tools, etc. It provides effective resources for children's online education and teachers' teaching. Outdoor experience courses are designed to attract children to participate. By recognizing animals and plants, understanding the growth process of crops, and learning agricultural production experience, we can improve children's quality in all aspects and achieve the purpose of children's cognitive education. In addition, the data collected by the system can help us better understand the basic situation of children for teachers, which is convenient for teachers to evaluate children and intervene in education.
6. Data module: the system will generate a large amount of data in the process of evaluating special children. The data module analyzes and integrates these data and generates corresponding charts from multiple angles and dimensions in an intuitive form, which is convenient for website users to view and use. At the same time, when the integrated data reaches a certain scale, it will also be conducive to the later big data analysis.

The article "Research on Children's Cognitive Education Based on Pathological Linguistics" was published in 2022. Journal: Occup Ther Int.

#### 2.3.3. Cognitive Presentation and Control of the Scene

The change of cognitive situation is conducive to children's cognitive generalization. Therefore, the system combines Agent technology with animation state machine. Realize the training situation change and control, and help children adapt to the situation change in the interaction. Agent refers to an Agent that can act autonomously. The system uses its intelligence to generate training content and give children feedback evaluation. Animation state machines are used to control and serialize animation. Each animation is called a state. In the generalization training game, after receiving the training request information, the Agent first queries the learning accuracy rate of each situation item in the database and generates the training order according to the principle of low training times and low accuracy item first. Then, associate the animation clip of each scene item to the motion of the corresponding state of the animation state machine in accordance with the order. Finally, the system initiates interactive tasks. According to the completion of tasks, the system gives feedback and evaluation of interactive operations to children in the form of voice and animation and automatically switches to the next scene for training, so as to control the changes of virtual scenes. After the training, save the answer information of each item into the database; the presentation and control flow of the cognitive scene is shown in Figure 4.

The core idea of the cognitive scene algorithm is to combine many weak classifiers with general classification ability into strong classifiers with strong ability. For each weak classifier, use the integral plot to quickly calculate the eigenvalues of the training samples, and calculate the error rate. The optimal weak classifier is selected according to the principle of the smallest error rate. The composition of the weak classifier is as follows:

(3) $$\begin{array}{c} R_{a}\left(b\right)=\left\{\begin{array}{c} 1,\;O_{a}T_{a}\left(b\right)\neq O_{a}\beta_{a},\\ 0,\;\text{others}. \end{array}\right. \end{array}$$

In the formula, *T*_*a*_ is the feature, *β*_a_ is the threshold, and *T*_*a*_ is the offset bit (value ± 1), so that the direction of the inequality is always the sign of inequality.

After that, new samples are added for a new round of training. After *N* rounds of iterations, the selected *N* optimal weak classifiers are combined into a strong classifier. The composition of the strong classifier is as follows:

(4) $$\begin{array}{c} R_{a}\left(b\right)=\left\{\begin{array}{c} 1,\;\overset{N}{\underset{n=1}{\sum }}O_{n}T_{n}\left(b\right)\geq 1.5\overset{N}{\underset{n=1}{\sum }}O_{n}{T_{n}}_{a},\\ 0,\;\text{others}. \end{array}\right. \end{array}$$

Finally, multiple strong classifiers are cascaded to obtain the final classifier that can be used for cognitive scenes.

### 2.4. Experimental Environment

This system is developed in Win10 and appropriate debugging in Linux and Win10. In the development process, the development tools used are Zendstudio10.6, SublimeText3, Postman, and Git. The business logic of the system adopts PHP language, and the overall technical architecture adopts domestic popular ThinkPHP3.2, and the program is developed iteration in MVC mode. The database uses Oracle's MySQL5.4; the front-end display layer uses Bootstrap V3.3.7 and uses the CDN acceleration service improved by Bootstrap. In the request mode, the use of Pjax not only improves user experience but also greatly reduces bandwidth consumption and server consumption. Eventually, the entire system will be deployed and run on Nginx servers. Experimental environment is shown in Table 3.

The article "Research on Children's Cognitive Education Based on Pathological Linguistics" was published in 2022. Journal: Occup Ther Int.

### 2.5. Evaluation Indicators

In the experiment, three indicators are used to analyze the data: contribution rate, the ratio of the data to the average, and the correct rate. The specific indicators have the following meanings.

#### 2.5.1. Contribution Rate

It is the ratio of the contribution of a single indicator to an outcome or process.

#### 2.5.2. Value to Average

It is the value as a percentage of the average or the value divided by the average multiplied by 100%.

#### 2.5.3. Correct Rate

It is the percentage of the correct number of the total, or the correct number divided by the total multiplied by 100%.

## 3. Results and Analysis

### 3.1. Dimension Analysis of Cognitive-Language Assessment

Based on pathological linguistics, a cognitive-language assessment database was established to further explore the characteristics of children's cognitive-language impairment. Through the dual-pass deep learning algorithm, the features in the two dimensions of speech flow and content flow are simultaneously extracted, so as to establish a correlation model between children's language and audio features, various annotation indicators, and language ability levels. Finally, the contribution rate of the six language dimensions is obtained. The six dimensions of verbal communication of 40 children with language impairment are shown in Figure 5, with different lines representing the scores of different subjects' verbal performance.

As can be seen from Figure 5, the contribution rates of the six language dimensions to the screening of children's language disorders also differ, among which fluency, voice, and capability rank the top three, with contribution rates of 29.6%, 25.7%, and 19.3%, respectively.

As shown in Figure 6, the contribution rates of various language indicators to verbal communication scores are also different. Among them, the top five language indicators are semantic, consonant sound mother, reducing language, content removal, and grammar.

At present, the data results annotated in the children's cognitive-language assessment database can be used as the training set of the model to further improve the accuracy of intelligent screening for language disorders. On the other hand, with the increase of the amount of children's speech data in different age groups, we have gradually established the norm of children's cognition-language assessment data, so as to more accurately assess the development of children's comprehensive speech ability, such as measuring children's language development age and clarifying the specific classification of language disorders. This is of great significance to the screening and diagnosis of children's language disorders and speech correction training.

The article "Research on Children's Cognitive Education Based on Pathological Linguistics" was published in 2022. Journal: Occup Ther Int.

### 3.2. An Intervention Analysis of Cognitive-Language Competence

The children's cognitive and speech evaluation system is mainly used in the study of special children's language ability; through careful comprehensive language competence evaluation, we can not only understand the words of the special children's development but also can be the special children's language dimension compared with normal children, targeted for their lifting scheme design of words. The labeled data of 120 children have been collected in this database, and the 6 special children are divided into 6 groups according to their actual ages for ANOVA univariate analysis. The results are shown in Figure 7.

The results showed that there were no significant differences in the scores of comprehensive language ability and six language dimensions among the six age groups (*P* > 0.05), indicating that age had no significant influence on the language ability of special children. The distribution of comprehensive language proficiency scores of these children is relatively scattered, indicating that the individual differences in language proficiency are large.

On the other hand, we refer to the average language scores of urban children of all ages and find that 58% of urban children aged 3-9 reach the average rate of comprehensive language proficiency scores. We compared the language scores of 35 special needs children aged 3-9 with those of urban children of the same age and found that only 40% of special-needs children reached the average language level of their age, which was defined as reaching the standard of language development. Specific data are shown in Table 4.

Different from that of normal children, special children's comprehensive language ability does not significantly improve with age. Of the 35 special children, the four year olds performed best, with 55.6 percent reaching the average language level for their age group. After the age of four, however, the performance of the special group declined relative to that of the same age group—the achievement rate got lower and lower with age.

In view of the fact that age has no significant influence on the language development of exceptional children, the relationship between the early intervention education and the comprehensive language ability score of exceptional children is further explored. We divided 90 subjects into three groups according to the age of early intervention education, including the intervention group before 3 years old, the intervention group between 3 and 6 years old, and the intervention group after 6 years old. The analysis of variance was conducted with the intervention age as the factor and comprehensive language ability score as the dependent variable. The results showed that early intervention significantly affected children's language development level (*F* = 3.484, *P* = 0.041 < 0.05). The scores of comprehensive language ability of the three groups of children with early intervention education are shown in Figure 8.

The article "Research on Children's Cognitive Education Based on Pathological Linguistics" was published in 2022. Journal: Occup Ther Int.

The test results showed that only the special children with early intervention education at the age of 3 had significantly better language development than the group at the age of 3-6. However, there was no significant difference between the children over 6 years old and the other two groups, which may be related to the fact that the children over 6 years old are generally older and get higher language scores accordingly. However, early intervention education before the age of 3 is beneficial to the language development of special children, which is basically consistent with previous studies. Therefore, for children with disabilities, early intervention education should be carried out as soon as possible to promote the language development of children.

### 3.3. Analysis on the Development of Cognitive Education

In order to evaluate the effect of cognitive education system and provide basis for further improvement, experimental tests are carried out in this paper. The experiment uses a different control group design; children with disorders are divided into intervention group and control group. Before starting the experiment, the two groups of children with disabilities completed the preexperiment assessment. After 10 weeks of intervention education, postexperiment evaluation was conducted. A total of 100 children with disabilities were recruited, including 53 males and 47 females, aged from 6 to 10 years, and divided into intervention group and control group with 50 children in each group. The intervention group and control group are shown in Table 5.

In view of the importance of language for cognitive education, the experimental results were recorded for a single indicator of language expression. After the experiment, the language cognition of children in the intervention group and the control group is shown in Figure 9.

Figure 9 shows the variation trend of the correct rate of word lingering, stress, and intonation in the intervention process. It can be seen that with the advance of intervention, the accuracy of word lingering, stress, and intonation has been significantly improved to a certain extent. The results showed that the correct rate of word lingering increased from 83.44% before intervention to 89.58% after intervention. The correct rate of stress increased from 41.23% before intervention to 56.25% after intervention. The correct rate of intonation increased from 67.01% before intervention to 78.13% after intervention. To sum up, we can see that after the intervention of language expression experimental teaching, the language expression of the subjects has been improved to a certain extent, and the accuracy of the use of various dimensions of language ability (phonemic construction, stress, phrase, and phrase continuity and intonation) has been improved.

The article "Research on Children's Cognitive Education Based on Pathological Linguistics" was published in 2022. Journal: Occup Ther Int.

Cognitive performance, cognitive generalization, emotional cognition, language expression, and hand-eye coordination were recorded before and after the experiment. The improvement of each index before and after education can be divided into three grades: 0 is ineffective, 1 is improved, and 2 is significantly effective. Before the assessment, the assistants were trained in assessment, and then parents and experts scored the improvement of children before and after education, and the assistants recorded and counted it. Data were processed by SPSS19.0 statistical software, measurement data were expressed as mean ± standard deviation, nonnormal distribution data were compared by a rank-sum test, and *P* < 0.05 was considered statistically significant. After the experiment, the cognitive education of children in the intervention group and the control group is shown in Figure 10.

As can be seen from Figure 10, the improvement degree of cognitive performance, cognitive generalization level, emotional cognition, and language expression in the intervention group was better than that in the control group, with statistical significance (*P* < 0.05). To sum up, using cognitive education system to intervene in children's cognition has largely improved children's cognitive level, which further shows that the evaluation and application effect of this system is very good.

## 4. Conclusion

Children are the future of the motherland and the hope of the nation. To escort the healthy growth of hundreds of millions of children, it is necessary to do a good job in children's cognitive education. Based on pathological linguistics, this study is aimed at constructing a comprehensive and effective evaluation and intervention system for children's cognitive education. The system includes a set of fixed guidance programs and accurate data annotation indicators. Based on the system, a database of cognitive-language development data of normal children and children with abnormal language is widely collected, and machine learning technology is used to realize the automatic assessment of children's cognitive-speech. At the theoretical level of pathology, intervention education for children's cognitive education is carried out based on six modules: user, assessment, scale, resources, teaching, and data. This system builds a platform for children's cognitive entity education, explores the cognitive development path of special children groups, and puts forward precise intervention education programs. The experiment proves that the language cognitive training model can effectively improve children's basic language ability and their cognitive ability to the surrounding things. The system is combined with a variety of intervention education methods to improve the effect of intelligence development, enhance children's cognitive ability to the greatest extent, and promote the healthy growth of children.

The article "Research on Children's Cognitive Education Based on Pathological Linguistics" was published in 2022. Journal: Occup Ther Int.

## Figures and Tables

**Figure 1:** Picture, video, and audio test diagram.

**Figure 2:** System architecture diagram.

**Figure 3:** Module diagram of cognitive education system.

**Figure 4:** Recognize the presentation and control flow of the scene.

**Figure 5:** Six-dimensional representation diagram.

**Figure 6:** Language index contribution rate chart.

**Figure 7:** Comprehensive language competence in six age groups.

**Figure 8:** Early intervention to educate children's comprehensive language ability.

**Figure 9:** Language cognition of two groups of children.

**Figure 10:** Cognitive education of children in intervention group and control group.

**Table 1:** Detailed labeling item table.

Item	Voice	Capability	Fluency	Grammar	Semantics	Logic
Label	Nonsensical mother error	Actual syllable number	Deed independent language	Grammatical errors	Semantic point cover	Logical error
			Argent			
	Tone error	Total time for pronunciation	Voice reconstruction times			
			Number of content removal			
	Master error	Speed	Repeat times			
			Number of pauses			
			Stunned			

Labeling method	Artificial labeling	Machine+artificial	Machine+artificial	Artificial labeling	Artificial labeling	Artificial labeling

**Table 2:** Database current overview table.

Age/year old	2-3	4	5	6	7-9	10-14	Total
The number of children is marked	73	114	129	112	148	62	638
Urban boy	32	43	50	35	60	12	232
Urban girl	37	32	33	26	66	10	204
Rural boy	10	32	30	35	86	77	270
Rural girl	11	30	33	45	65	76	260

**Table 3:** Experimental environment configuration.

System environment	Windows10	CentOS8.3	Windows Server2021
Server	Apache	Nginx	Apache
CPU	4.4GHz eight cores	4.4GHz dual -core	3.2GHz quad -core
RAM	16G	8G	128G
Hard disk	2T	1T	1T

The article "Research on Children's Cognitive Education Based on Pathological Linguistics" was published in 2022. Journal: Occup Ther Int.

**Table 4:** Special children language development level.

Generation	3	4	5	6	7–9	Total
Sample size	3	9	11	5	7	35
Number of people reaching the target	0	5	5	2	2	14
Compliance rat (%)	0	55.6	45.5	40	28.6	40

**Table 5:** Intervention group and control group data.

Grouping category	Intervention group	Control group
Number of people	50	50
Age (years)	8.13 ± 1.1	7.63 ± 1.2

## Data Availability

The data used to support the findings of this study are included within the article.

## References

[1] Bell-Dolan D., Wessler A. E. (1994). Attribution style of anxious children: extensions from cognitive theory and research on adult anxiety. *Journal of Anxiety Disorders*.

[2] Barolli L., Yim K., Chen H.-C. (2021). Innovative Mobile and Internet Services in Ubiquitous Computing:Proceedings of the 15th International Conference on Innovative Mobile and Internet Services in Ubiquitous Computing (IMIS-2021). *Springer Nature*.

[3] Babakr Z. H., Mohamedamin P., Kakamad K. (2019). Theory of cognitive development in children: a critical review. *Education Quarterly Reviews*.

[4] McGuire J. (2021). Australian early childhood educators and child cognition: a qualitative analysis using social cognitive theory. *Early Child Development and Care*.

[5] Opfer J. E., Kim D., Qin J. (2018). A cognitive theory of the state's influence on educational standards. *Language and culture in educational cognition*.

[6] Thojampa S. (2019). Social cognitive theories of child intervention in education: a discussion. *International Journal of Care Science*.

[7] Budi R. (2020). Using child cognitive theory to construct factors influencing primary and secondary practice: multi-level evidence from Maideen, East Java. *Journal of Health Promotion and Behavior*.

[8] Perales F., Baxter J. (2019). A matter of time: father involvement and child cognitive outcomes. *Journal of Marriage and Family*.

[9] Songco A., Hudson J. L., Fox E. (2018). A cognitive model of pathological worry in children and adolescents: a systematic review. *Clinical Child and Family Psychology Review*.

[10] BGrohmann M. K., Leivada E. (2018). Developmental, modal and pathological change - developmental and cognitive curves in patholinguistics. *Field of Psychology*.

[11] del Carmen Pamplona M., Ysunza P. A. (2019). The development history of speech cognitive correction for children with disabilities. *International Journal of Pediatric Sciences*.

[12] Bob J. (2018). Patholinguistics, education, and law: understanding language disorders in children and educational reform. *Pathological linguistics and Education*.

[13] Payne J. S. (2020). Developing L2 productive language skills online and the strategic use of instructional tools. *Foreign Language Annals*.

The article "Research on Children's Cognitive Education Based on Pathological Linguistics" was published in 2022. Journal: Occup Ther Int.

[14] Smithers L. G. (2018). Systematic review and meta-analysis of the effects of cognitive and health outcomes. *Natural Human Behavior*.

[15] Yulduz S., Maftuna A. (2021). The junior detective training program. *Romanian Society for Cell Biology*.

[16] Shulamit E. (2020). Language pedagogy for children's cognitive language development in bidirectional immersion schools. *Teacher ideology and practice*.

[17] Novak I., Honan I. (2020). Effectiveness of language cognitive education in children with disabilities: a systematic evaluation. *Australian Journal of Occupational Intervention therapy*.

[18] Grigorenko E. L. (2020). Understanding, educating, and supporting children with specific learning cognitive disabilities: 50 years of science and practice. *American Psychologist*.

[19] Thompson J. R., Walker V. L., Shogren K. A., Wehmeyer M. L. (2018). Expanding inclusive educational opportunities for students with the most important cognitive impairments through personalized support. *Intellectual and Developmental Disabilities*.

[20] Fiorello C. A., Wycoff K. L. (2018). Children's cognitive hypothesis testing: linking test results to educational interventions. *Cognitive Theory of Cognitive Children*.

